# Fatal Cervical Spinal Epidural Abscess and Spondylodiscitis Complicated With Rhombencephalitis Caused by Klebsiella pneumoniae: A Case Report and Literature Review

**DOI:** 10.7759/cureus.20100

**Published:** 2021-12-02

**Authors:** Nattapat Nitinai, Minth Punpichet, Worapong Nasomsong

**Affiliations:** 1 Department of Internal Medicine, Phramongkutklao Hospital and College of Medicine, Bangkok, THA; 2 Department of Radiology, Phramongkutklao Hospital and College of Medicine, Bangkok, THA; 3 Division of Infectious Disease and Department of Internal Medicine, Phramongkutklao Hospital and College of Medicine, Bangkok, THA

**Keywords:** brain abscess, klebsiella pneumoniae, rhombencephalitis, spondylodiscitis, spinal epidural abscess

## Abstract

Spinal epidural abscess (SEA) is a rare but sometimes life-threatening condition. The principal organisms in SEA and spondylodiscitis are gram-positive bacteria, e.g., *Staphylococcus* *aureus* and *Streptococci*. Spontaneous gram-negative SEA and spondylodiscitis especially *Klebsiella pneumoniae* are very rare. We report a 71-year-old Thai male with diabetes, presenting fever, enlarged neck mass, and progressive painful swallowing a week before admission. MRI of the whole spine demonstrated epidural abscess along the anterior thecal sac from C2 to C7 levels with spinal meningitis; multiple rim-enhancing lesions at the left sternocleidomastoid/levator scapulae, splenius capitis, semispinalis capitis, and bilateral scalene muscles; and rhombencephalitis with brain abscess. *Klebsiella pneumoniae* was isolated from blood culture. CT of the whole abdomen showed unremarkable intra-abdominal lesion. Intravenous ceftriaxone was administered, but the patient was unable to undergo surgical drainage due to unstable condition and died after two weeks of admission. Spontaneous SEA and spondylodiscitis caused by *K. pneumoniae* are very rare but sometimes fatal. In the case of SEA and spondylodiscitis, even when *K. pneumoniae* is uncommon, it should be also considered as a pathogen, especially when the patient had important risk factors.

## Introduction

Spinal epidural abscess (SEA) is a rare but severe condition and sometimes life-threatening. The incidence of SEA was 5.1 cases per 10,000 admissions, and bacteremia was the most common finding [1]. The typical clinical manifestations of SEA include fever, spinal pain, and neurological deficit, but all these features are presented in the late stage of the disease. A number of associated risk factors have been identified, including alcoholism, intravenous drug users (IVDU), diabetes mellitus (DM), and immunocompromised status [2]. SEA develops from three main mechanisms, including hematogenous spread from a distant source, adjacent organ spreading, and direct inoculation of microorganisms [3]. The major identified causative organism was *Staphylococcus aureus* and *Streptococci*, whereas identifiable gram-negative bacteria were far rarer in SEA [4]. *Klebsiella pneumoniae* are the family members of Enterobacterales, which are capable of causing various types of community-acquired and healthcare-associated infection (HAI), e.g., pneumonia, internal organ abscess, and bacteremia [5]. Currently, few cases have been reported with isolated and spontaneous *K. pneumoniae *SEA [6-14]. Here, we report the case of fatal isolate and spontaneous *K. pneumoniae* spondylodiscitis and SEA involving C1-C7 complicated with rhombencephalitis in a patient with diabetes.

## Case presentation

A 71-year-old Thai male presented to the emergency department with three days of progressively painful swallowing. Two weeks before admission, he reported soreness at both trapezii, shoulders, and scapular region. One week before admission, he developed a high-grade fever and then visited a private hospital, where he received cefdinir and clindamycin without any improvement. Three days before admission, he noticed an enlarged neck mass and experienced progressively painful swallowing.

His history was significant for stage III hypopharyngeal cancer with concurrent chemoradiation therapy and was in complete remission for two years. He presented coronary artery disease, well-controlled diabetes mellitus, and lumbosacral stenosis. He denied using herbal medication, smoking, and consuming alcohol, including illicit drug abuse.

On physical examination, his blood pressure was 130/58 mmHg, pulse rate 96/minute, respiratory rate 26/minute, and temperature 34.6°C. He presented a swollen left anterior neck erythema extending to the angle of the mandible and marked tenderness. Neurological examination was within the normal limit.

On the first day of admission in the intensive care unit (ICU), ceftriaxone was started due to positive blood culture from the private hospital report for *Klebsiella pneumoniae*. On the second day of admission, he developed progressive choking and hypoxemic cardiac arrest with successful resuscitation. He was in a stuporous condition, and his left-sided motor level was grade I. The initial blood test revealed a white blood cell count of 21,000/µL, comprising 96% neutrophils, a hemoglobin level of 9.1 g/dL, and a platelet level of 208,000/µL. AST was 61 IU/L, ALT was 64 IU/L, and ALP was 551 IU/L. MRI of the whole spine demonstrated epidural abscess along the anterior thecal sac from C2 to C7 levels with spinal meningitis; multiple rim-enhancing lesions at the left sternocleidomastoid/levator scapulae, splenius capitis, semispinalis capitis, and bilateral scalene muscles (Figures 1, 2); and rhombencephalitis with brain abscess (Figure 3). CT of the whole abdomen showed unremarkable intra-abdominal lesion.

**Figure 1:** Spondylodiscitis with epidural abscess, prevertebral abscess, and myelopathy. (A,B) Sagittal planes of T1WI, T2WI, and T1W FS with gadolinium enhancement sequences demonstrate abnormal T2 hyperintense signal change at the C5-C6 intervertebral disc (white arrow) as well as associated destruction of C5-C6 endplates, representing spondylodiscitis. Also, evidence of rim-enhancing T2 hyperintense signal anterior spinal epidural collection along the C2-C6 level (white arrowheads), representing spinal epidural abscess. The spinal epidural abscess causes compression of the cervical spinal cord at the C5-C6 level as well as abnormal T2 hyperintense change with multifocal patchy enhancement along the visualized spinal cord from the cervicomedullary junction to the T3 level (asterisk), likely compressive plus infectious myelopathy. (C) Evidence of prevertebral abscess at the C5-C6 level (black arrowhead).

**Figure 2:** Spondylodiscitis with epidural abscess and prevertebral abscess. (A,B) Axial planes of T2WI and T1W FS with gadolinium enhancement sequences at the C5-C6 level demonstrate rim-enhancing T2 hyperintense signal anterior spinal epidural collection (white arrowheads), representing spinal epidural abscess. The spinal epidural abscess compresses the cervical spinal cord at the corresponding level. Also, evidence of lobulated prevertebral abscess (black arrowhead) and left paravertebral abscess (white arrow). (C) Coronal T1W FS with gadolinium enhancement shows multifocal lobulated left paravertebral and intramuscular abscess at the left-sided cervical region (white arrow).

**Figure 3:** Rhombencephalitis with abscess. (A,B) Sagittal T1W and axial FLAIR with gadolinium enhancement at the posterior fossa demonstrate faint rim enhancement with T2/FLAIR hyperintense signal change at the medulla, including the obex, representing rhombencephalitis. (C,D) Axial DWI and ADC at the posterior fossa, and the content in the aforementioned rim-enhancing lesion at the medulla show restricted diffusion, which protrudes into the median aperture of the fourth ventricle, likely representing pus content.

In the first week of ICU admission, the patient still presented progressive quadriparesis (all extremities were grade I weak). The patient was unable to undergo surgical drainage of SEA due to unstable condition and a very high risk of surgery. The abscess at the left supraclavicular region was drained, and culture was sent for investigation. The hemoculture sent on the admission date was negative, and no organism was cultivated from the left scalenus muscle.

After two weeks of conservative therapy with ceftriaxone, he remained in a progressively debilitating condition. His motor power in all extremities comprised grade I, and his level of consciousness was comatose. Finally, he died after two weeks of admission.

## Discussion

Spinal epidural abscess is a rare but life-threatening condition. The most common causative pathogens are *S. aureus* and *Streptococci*. The concurrent adjacent spondylodiscitis commonly occurs owing to the contiguous spreading of microorganisms from the adjacent bone and disc, the most common route of infection [3,10]. Alcoholism, IVDU, diabetes mellitus, and immunocompromised status are the significant risk factors for SEA and spondylodiscitis [2]. Spontaneous gram-negative SEA and spondylodiscitis, especially *K. pneumoniae*, which often presents as a secondary infection from another organ and postneurosurgical conditions, remain very rare [11].

We performed an extensive literature search of the PubMed and Medline databases for articles published in English and identified only 10 case reports of *K. pneumoniae* SEA and four cases described as spontaneous SEA (Table 1). Among *K. pneumoniae* SEA cases, the classic manifestations of SEA, which included fever, spinal pain, and neurological deficit, presented. One-half of the patients presented with diabetes mellitus. The lumbar and thoracic spine are the major affected spinal levels; in contrast, only a few reports have described cervical SEA caused by *K. pneumoniae* as in the present case [9,13]. According to the clinical manifestations, this patient presented atypical features consisting of fever, neck mass, and painful swallowing with a lack of neurological deficit on admission. Interestingly, the progressive painful swallowing and choking later on the day might have reflected brain stem involvement from rhombencephalitis. However, the subsequently altered conscious level of the patient resulted from multiple factors including the progression of rhombencephalitis, hypoxic ischemic encephalopathy after cardiac arrest, and severe sepsis. In this case, an abdominal CT scan was performed to identify the primary focus of infection, revealing a normal result. Thus, we postulated that the spondylodiscitis and SEA in this patient may have occurred spontaneously associated with presumed silent bacteremia and consequently spread adjacent to the central nervous system [11]. To our knowledge, the present case constitutes the first case report of extensive spontaneous *K. pneumoniae* cervical SEA and spondylodiscitis complicated with rhombencephalitis resulting in a fatal outcome.

**Table 1:** Published cases of Klebsiella pneumoniae spinal epidural abscess.

Number	Age (year), sex, country	Positive culture	Affected spinal level	Underlying conditions	Clinical manifestations	Treatment	Outcome	Reference
1	71, male, Thailand	Blood	Cervical	DM, CAD, lumbar stenosis	Fever, neck mass, painful swallowing, paraparesis (spontaneous)	Antibiotics	Deceased	This case
2	56, male, Japan	Blood, pus	Thoracic	Hypertension	Fever and RUQ abdominal pain, liver abscess	Surgical and antibiotics	Improved	[14]
3	45, male, South Korea	Pus	Cervical	None	Neck pain, paresthesia, and weakness of the upper extremities (spontaneous)	Surgical and antibiotics	Improved	[13]
4	73, male, Taiwan	Blood	Thoracic	Intrahepatic duct stone	Fever, low back pain (spontaneous)	Antibiotics	Improved	[11]
5	74, female, Taiwan	Blood	Lumbar	L-infectious spondylitis/SEA s/p operation	Low back pain, radiating pain, paraparesis postneurosurgical	Surgical and antibiotics	Improved	[11]
6	75, female, Taiwan	Blood	Thoracicolumbar	DM, history of liver abscess	Fever, back pain, lung empyema, renal abscess, paraparesis, urine retention, UTI	Surgical and antibiotics	Improved	[11]
7	65, male, South Korea	Blood, pus	Lumbar	None	Fever and back pain, psoas abscess	Surgical and antibiotics	Improved	[7]
8	84, female, Portugal	Blood	Lumbar	Hypertension	Low back pain, fever (spontaneous)	Antibiotics	Improved	[6]
9	50, female, Malaysia	Pus	Lumbar	DM, history of severe lung infection	Fever, back pain, paraparesis, urine retention	Surgical and antibiotics	Improved	[10]
10	55, female, USA	Pus	Cervicothoracic	DM, hypertension	Fever, back pain, paraparesis, urine retention (spontaneous)	Surgical and antibiotics	Improved	[9]
11	65, male, China	Blood	Lumbar	After intestinal polypectomy	Back pain, limb numbness, weakness, fever	Surgical and antibiotics	Improved	[8]

The community-acquired *K. pneumoniae* in the present case was clinically suspected of hypervirulent *K. pneumoniae *(hvKP). hvKP infection often exhibited metastatic spread resulting in multifocal organ involvement and increased ability to involve the central nervous system and ocular regions [5]. hvKP infection tended to occur in younger, immunocompetent cases and caused more severe disease compared with classical *K. pneumoniae*. Diabetes mellitus is recognized as a significant risk factor in developing both SEA and hvKP infection [15]. hvKP infection is more frequently found among individuals from the community rather than HAI and is more common in the Asian Pacific Rim. The occurrence of *K. pneumoniae *SEA is mostly reported in Asia and possibly correlated with the hvKP strain (Table 1). Unfortunately, the isolated bacteria in this patient were discarded from the previous private hospital. Hence, neither molecular analysis nor string test to confirm hvKP strain was performed.

Among gram-negative SEA and spondylodiscitis, promptly combined therapy of both surgical drainage and antimicrobial therapy remains crucial [11]. Eight of 10 patients with *K. pneumoniae *SEA from related reports encountered favorable outcomes after combined surgical and medical therapy [7-10,13,14]. However, only two cases recovered after being conservatively treated with antibiotics [6,11]. Nevertheless, surgical drainage was limited because of unstable patient conditions, the extensive spreading of infection, and cardiac arrest from aspiration, which led to death.

## Conclusions

In conclusion, spontaneous SEA and spondylodiscitis caused by *K. pneumoniae* are very rare but sometimes fatal. Early diagnosis and prompt combined medical and surgical therapy constitute a considerable strategy. However, in the case of SEA and spondylodiscitis, uncommon organisms such as *K. pneumoniae* should also be considered, especially when important risk factors are established.
